The article "Is preoperative MRCP necessary for patients with gallstones? An analysis of the factors related to missed diagnosis of choledocholithiasis by preoperative ultrasound" was published in 2015. Journal: BMC Gastroenterol.

# Is preoperative MRCP necessary for patients with gallstones? An analysis of the factors related to missed diagnosis of choledocholithiasis by preoperative ultrasound

**DOI:** 10.1186/s12876-015-0392-1

**Published:** 2015-11-14

**Authors:** Yan Qiu, Zhengpeng Yang, Zhituo Li, Weihui Zhang, Dongbo Xue

**Affiliations:** Department of General Surgery, the First Affiliated Hospital of Harbin Medical University, 23 Youzheng St., Nangang Dist., 150001 Harbin, China

**Keywords:** Cholelithiasis, Diagnosis, Magnetic resonance cholangiopancreatography

## Abstract

**Background:**

The diagnosis of associated choledocholithiasis prior to cholecystectomy for patients with gallstones is important for the surgical decision and treatment efficacy. However, whether ultrasound is sufficient for preoperative diagnosis of choledocholithiasis remains controversial, with different opinions on whether routine magnetic resonance cholangiopancreatography (MRCP) is needed to detect the possible presence of common bile duct (CBD) stones.

**Methods:**

In this study, a total of 413 patients with gallstones who were admitted to the Department of General Surgery of the First Affiliated Hospital of Harbin Medical University in China for a period of 3 years and underwent both ultrasound and MRCP examinations were retrospectively analysed. After reviewing and screening these cases according to the literature, 11 indicators including gender, age, alanine aminotransferase, aspartate aminotransferase, total bilirubin, direct bilirubin, indirect bilirubin, alkaline phosphatase, γ-aminotransferase, CBD diameter, and concurrent acute cholecystitis were selected and comparatively analysed.

**Results:**

Among the 413 patients, a total of 109 cases showed concurrent gallstones and choledocholithiasis, accounting for 26.39 % of all cases. Among them, 60 cases of choledocholithiasis were revealed by ultrasound examination, accounting for 55.05 %, while 49 cases of choledocholithiasis were not detected by ultrasound examination but were confirmed by MRCP instead (the missed diagnosis rate of ultrasound was 44.95 %). The results of statistical analysis suggested that alanine aminotransferase, acute cholecystitis, and CBD diameter were the three most relevant factors for missed diagnosis by ultrasound.

**Conclusion:**

The accuracy of preoperative ultrasonography for the diagnosis of associated CBD stones for patients with gallstones is not high. However, elevated alanine aminotransferase, concurrent acute cholecystitis, and CBD diameter were identified as key factors that may affect the accuracy of the diagnosis. Thus, routine preoperative MRCP examination is suggested for patients with gallstones to rule out possible concomitant CBD stones.

The article "Is preoperative MRCP necessary for patients with gallstones? An analysis of the factors related to missed diagnosis of choledocholithiasis by preoperative ultrasound" was published in 2015. Journal: BMC Gastroenterol.

## Background

Cholelithiasis is a common disease requiring general surgery, in which gallstones account for the vast majority of procedures [1]. For patients with gallstones, approximately 5–15 % of cases are associated with choledocholithiasis [2–6]. With the development of medical technology, laparoscopic cholecystectomy (LC) has be more and more used for the treatment of gallstones [7]. However, during treatment, common bile duct stones are often easily overlooked. Thus, exploring an easy approach to preoperatively clarify the presence of associated CBD stones has important clinical implications.

Currently, patients with gallstones undergo ultrasonography examination and hepatobiliary biochemical serum analyses (bilirubin, alkaline phosphatase, etc.) as part of routine preoperative screening for CBD stones [8–16]. However, according to the literature, the accuracy and sensitivity of elevated liver enzymes in the diagnosis of choledocholithiasis are not high [12–16]. Due to the impact of intrahepatic bile duct stones, liver disease, and various sources of inflammation, acute short-term death of liver cells can result in the abnormal elevation of related predictors for choledocholithiasis, thereby affecting the diagnosis [2, 9, 10, 16]. Moreover, a large number of studies have indicated that the accuracy of ultrasound diagnosis of choledocholithiasis is not high [17–22]. When the specific hepatobiliary indicators evaluated in serum biochemical tests are abnormal, choledocholithiasis cannot be ruled out even if the ultrasound result is normal [20]. In particular, the accuracy of ultrasound is generally ranges from 55–65 % [17–23]. As a result, the diagnosis of choledocholithiasis by ultrasound and other conventional methods is not reliable.

In numerous preoperative imaging examinations, endoscopic retrograde cholangiopancreatography (ERCP) showed the highest accuracy in the diagnosis of choledocholithiasis, although this approach is invasive and expensive, with poor popularity [9, 10, 19, 24], so it is generally not a preferred option. The diagnostic accuracy of endoscopic ultrasound (EUS) for choledocholithiasis is similar to ERCP, but it needs special eqipments and skilled doctors [25]. Because some calculi cannot be analysed with computed tomography (CT), this approach is generally not used for the diagnosis of calculi [19, 26]. However, magnetic resonance cholangiopancreatography (MRCP) showed a high accuracy in the diagnosis of choledocholithiasis [22–24, 27]. In particular, Freitas ML reported that its accuracy is comparable to that of ERCP and IOC, and its sensitivity and specificity were shown to reach 95 % and 90 %, respectively [10, 19, 24].

The article "Is preoperative MRCP necessary for patients with gallstones? An analysis of the factors related to missed diagnosis of choledocholithiasis by preoperative ultrasound" was published in 2015. Journal: BMC Gastroenterol.

Among all approaches tested, MRCP has been considered an accurate and convenient method for the diagnosis of choledocholithiasis [17–24]. However, whether routine MRCP should be performed for patients with gallstones is considered controversial. Supporters of routine MRCP examination, including Ferrari FS, believe that its accuracy is comparable to that of ERCP and IOC and that it is a reliable tool for the diagnosis of choledocholithiasis [19]. In addition, Chang JH indicated that MRCP was the preferred examination method to assess CBD stones [22], and Maccioni F et al. reported that MRCP has great potential for development in the future and that it may play a valuable role and an alternative to ERCP in bile duct and pancreatic diseases [26]. On the other hand, the opponents of routine MRCP examination, such as Hoffmann C et al. believe that abdominal ultrasound is a highly efficient method for the preoperative diagnosis of gallbladder and CBD stones with high accuracy [28]. Karki S et al. reported that ultrasound was easy to operate, was non-invasive and served as a very valuable examination method for the diagnosis of obstructive jaundice caused by CBD stones [29]. Although the accuracy of choledocholithiasis diagnosis by MRCP has been clearly demonstrated, Epelboym I et al. indicated that, among the existing means of treatment, MRCP is expensive and inefficient and therefore not recommended as a preferred option [30]. Nebiker CA also stated that although MRCP plays a certain role in screening before gallstone surgery, it is not reasonable to routinely perform MRCP examination due to financial considerations [31].

Thus, it remains unclear whether limitations exist for ultrasonography to be used in the preoperative diagnosis of choledocholithiasis and whether routine MRCP is necessary in such cases. To answer these questions, the current study investigated the reliability of preoperative ultrasonography and the necessity of routine MRCP by performing a retrospective analysis with statistical methods.

## Methods

### Subjects

The participant information was anonymous and taken from the hospital database. This study was performed in accordance with the Helsinki II declaration and the approval for this study was obtained from the Committee for Medical Research Ethics of the First Affiliated Hospital of Harbin Medical University, which are the authority of research ethics in China.

A total of 413 patients with gallstones who were admitted to the Department of General Surgery of the First Affiliated Hospital of Harbin Medical University in China from January 1, 2011 to December 31, 2013 and underwent both ultrasound and MRCP examinations were retrospectively analysed. Of these patients, 109 met the criteria for this study and were included as subjects. The inclusion criteria consisted of a diagnosis of concurrent gallstone and choledocholithiasis, the administration of both ultrasound and MRCP examinations, and the presence of complete clinical data (complete medical record, liver function, MRCP, ultrasound, etc.). The exclusion criteria consisted of the absence of MRCP, lack of a choledocholithiasis diagnosis, liver disease or bile duct cancer, and a history of biliary tract surgery.

The article "Is preoperative MRCP necessary for patients with gallstones? An analysis of the factors related to missed diagnosis of choledocholithiasis by preoperative ultrasound" was published in 2015. Journal: BMC Gastroenterol.

### Patients grouping

Patients with gallstones who were admitted to the Department of General Surgery in our hospital for treatment were divided into two groups. Those with CBD stones revealed by both ultrasound and MRCP examinations, who were diagnosed as associated choledocholithiasis after subsequent clinical treatment, were included in the group defined as the ultrasonic detection group. Gallstone patients showing no obvious abnormalities in CBD revealed by ultrasound, with CBD stones revealed by MRCP examination, and who were diagnosed as associated choledocholithiasis after subsequent clinical treatment were included in the group defined as the ultrasound missed diagnosis group. This study evaluated a total of 109 gallstone patients with associated choledocholithiasis. The ultrasound missed diagnosis group included 49 cases of CBD stones that were revealed by MRCP but not ultrasound. In this group, 7 cases showed no corresponding clinical symptoms and presented normal laboratory examination results except for the MRCP examination; these patients were excluded due to the lack of relevant evidence for this study. Thus, the remaining 42 cases were included in the ultrasound missed diagnosis group. The ultrasound detection group included 60 cases. To perform comparative analysis with the ultrasound missed diagnosis group, 42 cases were randomly selected.

### Outcome measures

1. Gender: a categorical variable, male was presented as 1, and female was presented as 2.
2. Age: a counting variable, the age of the patient at admission was recorded and rounded up to the closest integer.
3. Indicators of liver function, including alanine aminotransferase (U/L), aspartate aminotransferase (U/L), total bilirubin (μmol/L), direct bilirubin (μmol/L), indirect bilirubin (μmol/L), alkaline phosphatase (U/L), and γ-aminotransferase (U/L): counting variables, the data from the first test of liver function after the patient was admitted to the hospital were recorded. Some patients had previously obtained laboratory data pertaining to liver function; those reference data that were considered valuable for diagnosis and treatment were recorded as reliable data.
4. Acute cholecystitis: a categorical variable, acute cholecystitis was recorded as 1, and no acute cholecystitis was recorded as 0.
5. CBD diameter: a counting variable, the data from the first MRCP examination after the patient was admitted to the hospital were recorded.

The article "Is preoperative MRCP necessary for patients with gallstones? An analysis of the factors related to missed diagnosis of choledocholithiasis by preoperative ultrasound" was published in 2015. Journal: BMC Gastroenterol.

### Statistical methods

All relevant data were statistically analysed using SPSS11.5 software. Different groups of data were analysed with appropriate statistical methods. For instance, counting data were compared using the chi-square test to detect if the difference was significant, while categorical data were compared using t-tests to detect whether the difference was significant. The significance level was set as α = 0.05. When *p* ≤ 0.05, the difference was considered statistically significant. Differences in data on relevant indicators were also analysed for significance. With univariate logistic regression analysis, the odds ratio (OR) and Wald value of each research factor of the 11 indicators were calculated, and those indicators showing statistical significance were selected. Then, further correlation analysis was carried out for the 11 indicators to select the indicators with statistically significant correlations with each other. Finally, correlation analysis was performed for the primary variable.

## Results

A total of 413 patients with gallstones who were admitted to the Department of General Surgery of the First Affiliated Hospital of Harbin Medical University in China from January 1, 2011 to December 31, 2013 and who underwent both ultrasound and MRCP examinations were retrospectively analysed. A total of 109 patients showed concurrent gallstones and choledocholithiasis, accounting for 26.39 % of all cases. Among these, 60/109 cases of choledocholithiasis were revealed by ultrasound examination, accounting for 55.05 %, while 49 cases showed no abnormality in the ultrasound examination. Seven cases showed normal results in the routine laboratory examination, with the exception of a CBD stone found by MRCP examination, accounting for 1.69 % of all cases and 6.42 % of the cases with choledocholithiasis.

### Analysis of the significance of the difference between the two groups of data using SPSS

#### Univariate logistic regression analysis

Univariate logistic regression analysis was carried out for the 11 indicators Table 1, and three indicators were found to be statistically significant (*p* < 0.05). These significant indicators included alanine aminotransferase, acute cholecystitis, and CBD diameter, as shown in Table 2.

**Table 1:** Univariate logistic regression analysis of the 11 indicators

No.	Indicator	Odds ratio (OR)	Wald value	*P* value
1	Gender	9.214 (1.363,62.285)	5.187	0.182
2	Age	1.015 (0.954,1.078)	0.214	0.192
3	Alanine aminotransferase	1.001 (0.992,1.009)	0.019	0.037
4	Aspartate aminotransferase	1.007 (1.000,1.014)	3.599	0.154
5	Total bilirubin	0.981 (0.868,1.108)	0.094	0.303
6	Direct bilirubin	1.019 (0.872,1.193)	0.058	0.454
7	Indirect bilirubin	0.976 (0.85 9,1.108)	0.145	0.760
8	Alkaline phosphatase	1.000 (0.997,1.003)	0.007	0.906
9	γ-aminotransferase	1.001 (0.998,1.004)	0.222	0.521
10	Acute cholecystitis	0.085 (0.012,0.599)	6.130	0.001
11	CBD diameter	0.017 (0.002,0.137)	14.705	0.001

The article "Is preoperative MRCP necessary for patients with gallstones? An analysis of the factors related to missed diagnosis of choledocholithiasis by preoperative ultrasound" was published in 2015. Journal: BMC Gastroenterol.

**Table 2:** Correlation analysis of the 11 indicators

	Gender	Age	Alanine aminotransferase	Aspartate aminotransferase	Total bilirubin	Direct bilirubin	Indirect bilirubin	Alkaline phosphatase	γ-aminotransferase	Acute cholecystitis	CBD diameter
Gender											
Age	−0.182 >0.05										
Alanine aminotransferase	0.111 >0.05	0.044 >0.05									
Aspartate aminotransferase	0.187 >0.05	0.022 >0.05	0.184 >0.05								
Total bilirubin	0.071 >0.05	−0.107 >0.05	0.278 <0.05*	−0.016 >0.05							
Direct bilirubin	0.073 >0.05	−0.201 >0.05	0.310 <0.05	0.005 >0.05	0.904 <0.05*						
Indirect bilirubin	−0.068 >0.05	0.072 >0.05	0.214 >0.05	0.010 >0.05	0.625 <0.05*	0.323 <0.05*					
Alkaline phosphatase	0.329 <0.05*	−0.024 >0.05	0.178 >0.05	−0.054 >0.05	0.086 >0.05	0.160 >0.05	−0.098 >0.05				
γ-aminotransferase	0.169 >0.05	0.021 >0.05	0.440 <0.05*	−0.018 >0.05	0.249 >0.05	0.283 <0.05*	0.087 >0.05	0.427 <0.05*			
Acute cholecystitis	0.243 >0.05	0.021 >0.05	0.221 >0.05	0.100 >0.05	0.155 >0.05	0.040 >0.05	0.073 >0.05	−0.015 >0.05	0.166 >0.05		
CBD diameter	0.011 >0.05	0.335 <0.05*	0.191 >0.05	0.319 <0.05*	−0.194 >0.05	−0.109 >0.05	−0.205 >0.05	−0.070 >0.05	−0.041 >0.05	0.065 >0.05	

*P < 0.05 indicates statistically significant correlation between the two indicators

#### Correlation analysis

To extend these results, correlation analysis was further performed for the 11 indicators. This analysis showed that *p* > 0.05 for all indicators, and the correlation coefficient <0.5, indicating no significant correlation, as shown in Table 3. The individual correlation analysis for the three indicators with significant differences between the two groups showed that, for these three indicators, *P* > 0.05 and the correlation coefficient <0.5, indicating no significant correlation, as shown in Table 4.

**Table 3:** Individual correlation analysis for the three indicators

	Alanine aminotransferase	Acute cholecystitis	CBD diameter
Alanine aminotransferase			
Acute cholecystitis	0.221>0.05*		
Common bile duct diameter	0.191>0.05*	0.065>0.05*	

*P > 0.05 indicates no statistically significant correlation between the two indicators

The article "Is preoperative MRCP necessary for patients with gallstones? An analysis of the factors related to missed diagnosis of choledocholithiasis by preoperative ultrasound" was published in 2015. Journal: BMC Gastroenterol.

**Table 4:** Correlation analysis for the primary variable (missed diagnosis of choledocholithiasis by ultrasound)

	Alanine aminotransferase	Acute cholecystitis	CBD diameter
Primary variable (missed diagnosis of choledocholithiasis by ultrasound)	0.277	0.360	−0.624
*P* value	0.038*	0.001*	0.000*

*P < 0.05 indicates statistically significant correlation between the indicator and the primary variable

#### Correlation analysis for the primary variable

Correlation analyses for the three indicators with significant differences between the two groups and the primary variable were carried out. These results showed that alanine aminotransferase and acute cholecystitis were positively correlated with the primary variable, while the diameter of the CBD was negatively correlated with the primary variable. In other words, higher levels of alanine aminotransferase were associated with an increased likelihood of missed diagnosis of choledocholithiasis by ultrasound. In addition, the likelihood of missed diagnosis of CBD stones by ultrasound was higher in patients with acute cholecystitis, and CBD diameters closer to normal were associated with a greater likelihood of missed diagnosis of CBD stones by ultrasound, as shown in Table 4.

## Discussion

Cholelithiasis is a common disease requiring general surgery, and due to the rapid development of medical technology, its diagnosis and treatment have gradually matured. However, the biliary system is extremely complex, and there remains no standard for the diagnosis of cholelithiasis.

In this study, information pertaining to patients with concurrent gallstones and choledocholithiasis was collected and analysed to investigate the reliability of ultrasound in the diagnosis of concurrent gallstones and choledocholithiasis, as well as the necessity of routine MRCP. Retrospective analysis of the collected cases showed that, among a total of 413 patients with gallstones who were admitted to the Department of General Surgery of our hospital within 3 years and underwent both ultrasound and MRCP examinations, 109 cases showed concurrent gallstones and choledocholithiasis, accounting for 26.39 % of all cases. Among these, 60 cases of choledocholithiasis were revealed by ultrasound examination, with a detection rate of 55.05 %, while the remaining 49 cases of choledocholithiasis were not detected by ultrasound examination (the missed diagnosis rate of ultrasound was 44.95 %). The above conclusion suggests that ultrasound is not a reliable method for the preoperative screening of CBD stones.

By reviewing the literature, 11 observation indicators were selected for further analysis. The statistical baseline description and analysis of the differences between the two groups showed that three indicators, including alanine aminotransferase, acute cholecystitis, and CBD diameter, were significantly different between the two groups. In addition, univariate logistic regression analysis for the 11 indicators showed that these three indicators were statistically significant, and correlation analysis for these three indicators with statistical significance showed no statistically significant correlation between them. In particular, the correlation analysis for these three indicators and “ultrasound missed diagnosis of CBD stones” as the primary variable showed that alanine aminotransferase and acute cholecystitis were positively correlated with the primary variable, while CBD diameter was negatively correlated with the primary variable.

The article "Is preoperative MRCP necessary for patients with gallstones? An analysis of the factors related to missed diagnosis of choledocholithiasis by preoperative ultrasound" was published in 2015. Journal: BMC Gastroenterol.

Regarding the hepatobiliary indicators of serum biochemistry, the levels of bilirubin and alkaline phosphatase are considered to be significantly related to CBD stones. In recent years, γ-aminotransferase has attracted increasing attention, with a level greater than 90 U/L considered a risk factor for CBD stones [8, 10, 15, 16, 32, 33]. In this retrospective study, the levels of bilirubin, alkaline phosphatase, and γ-aminotransferase in the two groups of subjects were significantly increased, suggesting that they are closely related to the occurrence of CBD stones. However, these three indicators were not significantly different between the two groups. Regarding the relationship between alanine aminotransferase and CBD stones, few relevant studies are available in the literature, mainly due to poor specificity. Padda MS et al. reported that alanine aminotransferase, alkaline phosphatase, and CBD diameter are important for the diagnosis of concurrent gallstones and CBD stones [13]. Similarly, Sharara AI et al. found that elevated alanine aminotransferase and aspartate aminotransferase levels were related to the timing of the pain caused by CBD stones [34]. To date, the relationship between the alanine aminotransferase level and an ultrasound missed diagnosis of CBD stones has not been reported. Considering the limitations of this study, the relationship between alanine aminotransferase and ultrasound missed diagnosis of CBD stones remains poorly defined.

The relationship between acute cholecystitis and CBD stones had been reported in many studies, with many reports showing acute cholecystitis to be a significant clinical symptom of choledocholithiasis. Tsai TJ et al. reported that acute cholecystitis is one of the severe concurrent complications of the recurrence of choledocholithiasis after treatment [35], and Boys JA et al. indicated that, in the case of choledocholithiasis associated with acute cholecystitis, the diagnosis of CBD stones based on the CBD diameter by ultrasound is not reliable [35]. Acute cholecystitis can cause significant clinical symptoms, but because of its rapid development, the body quickly responds to stress, leading to significant changes in the value of certain indicators, thereby masking the CBD stones. Wong HP et al. proposed that MRCP is the best method to diagnose acute cholecystitis associated with choledocholithiasis [9], and Lee JK et al. indicated that the CBD diameter and bilirubin level were related to the development of acute cholecystitis. It is generally agreed that there is a relationship between the occurrences of acute cholecystitis and choledocholithiasis, although no relationship between acute cholecystitis and a diagnosis of choledocholithiasis missed by ultrasound has been reported [33]. Although this study confirmed the relationship between these variables using statistical methods, the mechanism for how acute cholecystitis affects the ultrasound diagnosis of choledocholithiasis remains unclear, and further investigation is needed.

The article "Is preoperative MRCP necessary for patients with gallstones? An analysis of the factors related to missed diagnosis of choledocholithiasis by preoperative ultrasound" was published in 2015. Journal: BMC Gastroenterol.

In contrast, the relationship between CBD diameter and CBD stones is more clear, as a larger CBD diameter is one of the major risk factors for CBD stones. However, a large number of studies have shown that the diameter of the CBD is not positively correlated with the occurrence of CBD stones [36–38]. For instance, the study by Isherwood J et al. showed that only 37 % of patients with choledocholithiasis presented a widened CBD diameter on ultrasound. In addition, these authors suggested that if the indicators of liver function related to choledocholithiasis are abnormal, choledocholithiasis must be further excluded even if the ultrasound shows a normal CBD diameter [20]. Laing FC et al. demonstrated that at least 30 % of CBD stones showed no dilatation of CBD, and ultrasound was unable to diagnose these patients, which was likely affected by many factors [21]. Wong HP et al. also indicated that the correlation between CBD diameter and associated CBD stones was not as strong as previously thought, as ultrasound can only provide data limited to the CBD area, with only a limited ability to directly measure the diameter of a CBD stone [9]. In addition, Karvonen J reported that the CBD diameter did not predict the progression of CBD stones [39]. The problems addressed in the above studies are consistent with the findings of our study; a nearly normal CBD diameter did not reflect the absence of CBD stones, which may easily mislead physicians and result in the missed diagnosis of CBD stones.

The article "Is preoperative MRCP necessary for patients with gallstones? An analysis of the factors related to missed diagnosis of choledocholithiasis by preoperative ultrasound" was published in 2015. Journal: BMC Gastroenterol.

At present, MRCP, ERCP, EUS, intraoperative cholangiography and intraoperative choledochoscopy are the effective methods for diagnosis of choledocholithiasis [26, 28, 40, 41]. Ainsworth AP et al. [41] and Meagher et al. [42] considered that ERCP advantaged in the diagnosis of common bile duct diseases. ERCP is a traumatogenic examination that required professional hospital equipment so it is not fit for screening a large number of patients. However, MRCP is a nontraumatogenic examination that can be finished in one day before the operation and the average cost of the examination is 88 dollars in China. More over, MRCP has no obvious effect on the cost of patients and the length of hospital stay. So, MRCP is a feasible examination of screening the suspected choledocholithiasis patients and it could bring the economic benefit. Morris S et al. [40] considered ERCP, compared to MRCP and EUS, was the most effective diagnostic methods of choledocholithiasis through analyzing the sensitivity of the examinations, the average cost and quality of life. However, Vergel YB et al. [43] considered MRCP was better than ERCP in saving the cost and improving patients’ postoperative quality of life for the suspected choledocholithiasis patients through comparing with each other.

Among the cases included in this study, 7 cases showed normal results for routine laboratory examinations, with the exception that a CBD stone was revealed by MRCP examination, accounting for 1.69 % of all cases and 6.42 % of the cases with choledocholithiasis. This strong concealment may lead to serious consequences, and although its proportion was as low as 1.69 % of all cases, the resulting problem can not be ignored.

Based on this study, the importance of preoperative MRCP examination was clearly demonstrated. This approach is convenient and accurate, non-invasive and safe. With increasing economic development and attention on public health, the cost of MRCP examination should be acceptable.

Epelboym I, Nebiker CA, who believe that because of the economic burden caused by MRCP, MRCP is not recommended for choledocholithiasis preferred to be checked [31, 32]. However, after the above discussion, we can not be ignored that MRCP has its advantages in screening patients with suspected choledocholithiasis in. This article does not investigation and analysis cost effective for patients. However, according to a basic understanding of the Chinese MRCP average cost of 350 yuan, with an average economic comparison of China’s national conditions and the world, with MRCP gallstone patients with suspected choledocholithiasis screening is feasible in economic benefits.

The article "Is preoperative MRCP necessary for patients with gallstones? An analysis of the factors related to missed diagnosis of choledocholithiasis by preoperative ultrasound" was published in 2015. Journal: BMC Gastroenterol.

## Conclusion

The accuracy of preoperative ultrasonography in the diagnosis of patients with concurrent gallstones and CBD stones is not high. In particular, elevated alanine aminotransferase, acute cholecystitis, and nearly normal CBD diameters were identified as key factors that may affect the accuracy of its diagnosis. Thus, routine preoperative MRCP examination is recommended for patients with gallstones to rule out the likelihood of concomitant CBD stones.
